The article "Design of Multimodal Neural Network Control System for Mechanically Driven Reconfigurable Robot" was published in 2022. Journal: Comput Intell Neurosci.

# Design of Multimodal Neural Network Control System for Mechanically Driven Reconfigurable Robot

**DOI:** 10.1155/2022/2447263

**Published:** 2022-05-25

**Authors:** Zhang Youchun, Zhang Gongyong

**Affiliations:** ^1^School of Application Engineering, Anhui Business and Technology College, Hefei 231131, China; ^2^School of Electrical Engineering, Binzhou University, Binzhou 256600, China

## Abstract

According to the characteristics and division rules of the modules, this paper divides the rotary module, the swing module, and the mobile module. In order to realize the rapid identification of modules, according to the basic principles of module design, the above modules are put into the module library established by Access. According to the modular modeling method, kinematic models are established, respectively. In order to automatically establish the kinematic model of the robot, a unified expression of modules is established. According to the unified expression of the modules, the kinematics of the reconfigurable robot is analyzed. According to the characteristics of the configuration plane, the configuration plane is divided, and the expression form of the position and attitude of the configuration plane is given. Combined with the principle of neural network and multimodal information fusion, a multimodal information fusion model based on long- and short-term memory neural network is established. Aiming at the control problem of mechanically driven reconfigurable robots, a specific long- and short-term memory neural network model is designed, and the long- and short-term memory neural network algorithm is applied to the robot control problem based on multimodal information fusion. The design of the controller and driver of each joint is the basis of the distributed control system. This paper discusses the hardware design of the joint controller and driver and the realization of the position control system and discusses the method of realizing distributed control based on the Modbus protocol of RS485 communication. Through the comprehensive experiment of the configuration, the point control and the continuous path control are carried out to verify the correctness of the theoretical analysis of the system and the reliability of the system hardware and software operation.

## 1. Introduction

Traditional robots are developed for specific application tasks [1]. Although some different tasks can be completed through programming, the scope of tasks that can be completed is limited due to the limitation of their own structure. In modern robot applications, the tasks are complex and changeable, and the operating ability of the robots used is required to adapt to changes in the environment and tasks [2]. For this reason, the concept of reconfigurable robots is proposed. A reconfigurable robot is composed of many modules with different functions. Using these modules, robots of different configurations can be quickly combined, but this combination is not a simple mechanical assembly [3]. The reconstructed robot will be able to adapt to different working environments and tasks, with good flexibility.

The article "Design of Multimodal Neural Network Control System for Mechanically Driven Reconfigurable Robot" was published in 2022. Journal: Comput Intell Neurosci.

The reconfigurable robot systems that have been developed are generally divided into two categories: static reconfigurable robots and self-reconfigurable robots [4]. The static reconfigurable robot completes the configuration change through manual assistance, while the self-reconfigurable robot automatically changes the connection relationship of each module according to the changes of the working environment and tasks, so as to realize the configuration reconfiguration [5]. For example, a snake-shaped reconfigurable robot is a self-reconfigurable robot. When passing through a narrow field, it maintains a snake-like configuration, and when it is on a flat ground, it changes its configuration and reconfigures into a multilegged walking robot.

The reconfigurable modular robot is composed of a series of intelligent modules with interchangeability that can be connected to each other and can be reconfigured into robots with different topological structures according to the task requirements [6]. On the basis of modular robot research, it uses link and joint modules of different performance sizes to form a specific robot configuration. Furthermore, modularization makes the dimensions and specifications of various functional components of the robot unified, and the unit modules of the same component have the same structure and function [7]. The standard parts suitable for large-scale industrial production greatly improve the production efficiency, the compatibility of the robot system and the automatic repair power of the robot, and the most important thing is to greatly reduce the design and production costs. In modern industry, the commercialized modular joint itself is an intelligent unit integrating communication, control, drive, and transmission [8]. Therefore, in terms of saving weight, saving space, and increasing robustness, the characteristics of the reconfigurable robot have a high degree of conformity with the actual needs and can change its configuration according to the task requirements to complete tasks in unknown environments and unknown requirements [9,10].

In this paper, the reconfigurable robot modules are divided into several types, and a reconfigurable robot module library is established according to each module according to its characteristics and parameters, which is used to find and select the required robot module types and parameters. And according to the difference of each module, the kinematic model of each module and a unified kinematic model that can be established automatically are established. In this paper, long- and short-term memory neural network is used to fuse multimodal information. The basic principle of long- and short-term memory neural network and the method of robot control using long- and short-term memory neural network for multimodal information fusion are introduced in detail. This paper discusses the hardware design of the control part of the reconfigurable modular robot system. Based on the PID controller with Anti-windup correction, a single-joint position control with velocity loop and position loop PID is designed. The control program and interface of the host computer are designed, and the Modbus communication protocol based on RS485 is used to realize the distributed control of the host computer and each joint controller [11]. Finally, experiments with various configurations are carried out, and the results of point control and continuous path control experiments of two-DOF and six-DOF configurations are given, which verify the validity and reliability of the software and hardware of the system.

The article "Design of Multimodal Neural Network Control System for Mechanically Driven Reconfigurable Robot" was published in 2022. Journal: Comput Intell Neurosci.

## 2. Related Work

Relevant scholars have designed a module library, studied the design of the configuration and the analysis methods of kinematics and dynamics, and developed a variety of reconfigurable systems, including a seven-degree-of-freedom arm, a six-degree-of-freedom three-parallel manipulator, and a three-degree-of-freedom manipulator [12]. The control method used for the reconfigurable robot is also adaptable to modularization. Each module is designed with an independent controller. The communication method adopts the CAN bus method. The PC is used as the host computer. Through the CAN bus, each module can be identified and controlled to achieve coordination [13].

Related scholars start from obtaining the geometric representation of the model configuration and completely consider the process of closed-form dynamic equations; first, an information storage matrix AIM is proposed to record the relationship between the geometric topology and the modules of the robot [14]. The model is obtained from AIM. After the required information of the model is obtained, the iterative Newton-Euler algorithm is used to automatically generate the dynamic equation of the corresponding configuration of the robot [15]. Scholars proposed an automatic generation method of dynamic equations, which can represent the relationship between the joint angular velocity, angular acceleration, and force/torque of each module and completes the automatic modeling of reconfigurable robots through compensation iteration method [16].

The article "Design of Multimodal Neural Network Control System for Mechanically Driven Reconfigurable Robot" was published in 2022. Journal: Comput Intell Neurosci.

The sliding mode variable structure controller realizes variable structure control by establishing a sliding model on the switch surface. At this time, the system is not sensitive to the parameters and external disturbances, so only the range of the parameters is needed and the precise dynamic model is not needed. However, the sliding mode variable structure has the above advantages, but also has the significant defects that the uncertain interference must meet the matching conditions and the chattering phenomenon is serious.

In the common sliding mode variable structure controller, the third-order derivation of the angle control variable is required, which makes the control law derivation process cumbersome and complicated. The combination of sliding mode variable structure control design and other control methods is the direction of further research on sliding mode variable structure controller, and this combination often further increases the tediousness and complexity of the control law [17,18]. In recent years, due to the ability of artificial neural network to approximate any nonlinear mapping through learning, most literature use neural network to approximate the entire robot dynamics model, and the other type uses neural network to compensate for the uncertainty of the model [19].

Relevant scholars introduced deep learning into the feature extraction of multimodal data, integrated two different information modalities of audio and video on speech recognition data, and trained a deep belief network to extract joint feature expressions from the two modalities, which has achieved good results in the video semantic understanding task [20].

Relevant scholars have applied deep neural network to image retrieval tasks, using various features extracted from image data as image modalities, and image text annotations made by users as text modalities, constructing the same deep neural network model [21,22]. These two modalities are simultaneously trained to obtain a joint high-level abstract semantic feature for image classification and retrieval, which also achieves good results. However, these models do not take into account that the importance of different modalities for the current learning task is not the same and only focus on how to effectively use multiple modalities for feature extraction at the same time, without involving the selection of modalities and harmful modalities filter. Due to the intermodal heterogeneity of multimodal data itself, most applications of multimodal data focus on using multimodal data to build models separately, and then fuse them in decision-making [23].

The article "Design of Multimodal Neural Network Control System for Mechanically Driven Reconfigurable Robot" was published in 2022. Journal: Comput Intell Neurosci.

## 3. Methods

### 3.1. Division of Reconfigurable Robot Modules

The reconfigurable robot should have the characteristics that it can be directly replaced or connected in order to achieve the required configuration, then the reconfigurable robot should be able to realize the standardization of electrical or mechanical interfaces, not only functional independence but also unified input. The robot modules with different functions can be directly connected to complete the desired task [24].

The module itself of a modular robot should have the following basic characteristics, which play an important role in robot mechanical manufacturing.

1. Independence of modules: the reconfigurable robot system is composed of each subsystem, and each subsystem has different functions. Therefore, it is often hoped that each module has independent characteristics, which reduces the coupling of the robot modules. .
2. Universal standard interface: modular robots need to have consistent electrical and mechanical interfaces because they can continuously change configurations to meet their mission requirements, making it very convenient to replace modules, and their functional interfaces can be quickly changed.
3. The module should be able to complete the overall configuration of the robot and exist: although the robot module can be regarded as an independent individual, it is also based on the entire robot configuration and completed functions, so it should be independent while satisfying its independence.
4. Modules should be able to have different levels according to their characteristics: each independent module is combined into a submodule with the same function, and each module together constitutes a parent module, which divides the modules into different levels. The control of the module can complete different functions.

This paper mainly adopts the division form of connection module and single degree of freedom module. In order to realize the changeable configuration of the reconfigurable robot, the connection module can not only play the role of connecting each module but also have the characteristics of adjusting the center of each joint, and the single-degree-of-freedom module is mainly the basic module.

### 3.2. Kinematic Modeling of Reconfigurable Robot Modules

In order to carry out further research on the reconfigurable robot, it is necessary to establish its kinematic model first. The generalized transformation matrix method is generally used for the traditional configuration of the robot, but this kind of robot is mainly based on the open-chain structure. The continuous change of the reconfigurable robot configuration makes it impossible to determine the end pose matrix of the robot module even if a previous module is selected, so this method is often not used.

The article "Design of Multimodal Neural Network Control System for Mechanically Driven Reconfigurable Robot" was published in 2022. Journal: Comput Intell Neurosci.

The D-H method can determine the kinematic equation through four parameters, but the parameters are difficult to determine. The derivation of the exponential product formula is very complicated. Considering many factors, this paper deduces the expression of a unified mathematical model by establishing models for the rocking module, the moving module, the connecting module, and the slewing module, and the kinematics model can be solved automatically by given parameters.

#### 3.2.1. Modeling of the Rocking Module

The origin of the rocking module is set as the center point of the upper and lower contact surfaces. The coordinate origin of the rocking module has no displacement change with the previous rocking module. The rocking of the rocking module mainly depends on the relative rotation of the next rocking module. The two coordinate systems on the connecting surface of the rocking module are mainly represented by standard coordinates, and their mathematical models are deduced. The modeling expression of the rocking module is

(1) $$\begin{array}{c} T_{\text{yb}}=\left[\begin{array}{cccc} -1 & 1 & \sin\;\beta_{\text{yb}} & -\cos\;\beta_{\text{yb}}\\ 1 & -h_{\text{yb}}\sin\;\beta_{yb} & h_{\text{yb}}\cos\;\beta_{\text{yb}} & -1\\ \cos\;\beta_{\text{yb}} & -\sin\;\beta_{\text{yb}} & 0 & 1\\ 0 & 1 & -1 & \sin\;\beta_{\text{yb}} \end{array}\right]. \end{array}$$

In the formula, *β*_*yb*_ is the upper and lower twist angle of the rocking module; *h*_*yb*_ is the distance between the origin of the rocking module and the contact surface of the adjacent connected modules.

#### 3.2.2. Modeling of the Rotary Module

The lower half of the slewing module remains stationary, and its coordinate system is established at the connection between the upper half and the lower half of the slewing module, and the relative rotation of the upper half causes the relative change between the coordinate systems. The modeling expression of the rotary module is

(2) $$\begin{array}{c} T_{\text{hz}}=\left[\begin{array}{cccc} \sin\;\theta_{\text{hz}} & -1 & \cos\;\theta_{\text{hz}} & -l_{\text{hz}}\\ 0 & 1 & 0 & 1-\cos\;\theta_{\text{hz}}\\ -\cos\;\theta_{\text{hz}} & -1 & 1-\sin\;\theta_{\text{hz}} & 1\\ l_{\text{hz}} & 0 & 1-\cos\;\theta_{\text{hz}} & -\sin\;\theta_{\text{hz}} \end{array}\right]. \end{array}$$

In the formula, *θ*_*hz*_ is the torsion angle of the upper and lower parts of the rotary module; *l*_*hz*_ is the distance between the rotary and the center of the adjacent connected modules.

The article "Design of Multimodal Neural Network Control System for Mechanically Driven Reconfigurable Robot" was published in 2022. Journal: Comput Intell Neurosci.

#### 3.2.3. Modeling of Mobile Modules

The upper half of the mobile module does not move, and the origin is set at the two connecting surfaces. The change between the coordinate systems of the mobile module is mainly through the relative rotation of the lower half of the mobile module. The upper and lower parts are mainly composed of standard components.

The mobile module modeling expression is

(3) $$\begin{array}{c} T_{\text{yd}}=\left[\begin{array}{cccc} -1 & h_{\text{yd}} & 0 & -1\\ 1 & -H_{\text{yd}} & -1 & 0\\ h_{\text{yd}} & 0 & H_{\text{yd}} & 0\\ 1 & 0 & 0 & -h_{\text{yd}} \end{array}\right]. \end{array}$$

In the formula, *H*_*yd*_ is the distance between the origin of the mobile module and the center of the adjacent connected modules; *h*_*yd*_ is the movement amount of the mobile module.

#### 3.2.4. Unified Expression of Modules

In order to realize that the kinematic model can be automatically established with given parameters, a unified modeling expression *ξ* is derived:

(4) $$\begin{array}{c} \xi =\left[\begin{array}{cccc} 1-\sin\;\theta \;\cos\;\beta & 1 & h\;\sin\;\beta & -\cos\;\beta \\ 1 & -h\;\sin\;\beta & 0 & -1\\ \cos\;\beta & 1-\sin\;\beta & h\;\cos\;\beta \;\sin\;\theta & l-w\\ -1 & 0 & -1 & 1-h\;\sin\;\theta \end{array}\right]. \end{array}$$

The parameter has a value when the parameter is the parameter of the specified module, and the value of the parameter unrelated to the module is zero. When the specified module is a rotary module, *θ* is the torsion angle of the upper and lower parts; when the specified module is a swing module, *β* is the relative swing angle of the upper and lower parts, and *h* is the relative distance between the upper and lower parts; when the module is rotated, *l* is the connection length; when the specified module is a moving module, *w* is the relative movement value.

### 3.3. Establishment of Reconfigurable Robot Module Library

Because there are many kinds of modules and they are used more frequently, by establishing a module library of the robot, users can check the specific parameter information of each module more intuitively without having to search manually, so as to quickly find the type of module they need, or they can also find the required module type according to their needs. We put the following information such as basic modules or connection modules into the module library and also put its specific dimensions such as radius, weight, and height into the module library. Drive capacity, speed, torque, and other information should also be placed in the module library. And the established module library can not only store information but also can directly add information and types of new modules through a simple button, which is convenient for finding module information and has the feature of deleting module information [25].

The article "Design of Multimodal Neural Network Control System for Mechanically Driven Reconfigurable Robot" was published in 2022. Journal: Comput Intell Neurosci.

The module library of the established reconfigurable robot can find out the type of module after giving simple information and provides a simple search method. Information such as size, weight, torque, speed, and other information are put into a database together to facilitate the completion of kinematics and dynamics solution, workspace solution and the corresponding initialization of trajectory planning, and more quickly find the ones that meet the conditions.

You put the joint information of the reconfigurable robot into the Access database, display all the selections in the form of a table, display the selected information at the top, and add the records of the Access database through the programming of VC++. After clicking OK, a dialog box will pop up to display the selected information and confirm it. After completing the selection of a joint, it will appear in the main interface.

### 3.4. Design of Long- and Short-Term Memory Neural Network

In a long-term memory neural network, the hidden layer consists of memory blocks, which are considered as neurons of the hidden layer, as shown in Figure 1.

Memory blocks add or delete information from neuron states through structures called gates. The key part of the memory block is the gate structure. The gate structure controls how much information is passed.

Each memory block is associated with an input gate, an output gate, and an internal state fed into itself across time. In this model, for each memory cell, three sets of weights are trained from the input, including the complete hidden state from the previous time step, one fed to the input node, one to the input gate, and one to the output gate. The most central node in the cell is called the memory and is fed back to itself with a weight of one across time. The self-connecting edge of the memory is called the constant error carousel.

Input gates, output gates, and forget gates all accept activation values from inside and outside the memory block and control the state of the memory. The activation function *f* of the gate structure uses the sigmod function, so the activation value is between 0 and 1, 0 means the door is fully closed, 1 means the door is fully open, and intermediate values indicate how open the door is. The memory input and output activation functions g and *h* use the tanh function. Lookout connections lead from memory to individual gate structures. The observation hole connection is weighted, and the remaining connections in the memory block have no weight (or the weight is fixed at 1).

The article "Design of Multimodal Neural Network Control System for Mechanically Driven Reconfigurable Robot" was published in 2022. Journal: Comput Intell Neurosci.

During forward propagation in a memory block, the input gate learns to decide when to let activations pass into the memory cell, and the output gate learns when to let activations go out of the memory cell. Correspondingly, during backpropagation in the memory block, the output gate is learning when to let errors flow into the memory cell, and the input gate is learning when to let it flow out of the memory cell and on to the rest of the network [26].

Multiple memory blocks are used as hidden layer neurons, which together constitute the recurrent layer of the long- and short-term memory neural network. We can construct a long- and short-term neural network model suitable for the actual problem according to the actual problem. In the recursive layer, the neurons of each memory block are connected to each other to form a complex recursive network structure.

In general, from the output layer to the hidden layer, we can calculate it according to the following formula:

(5) $$\begin{array}{c} a_{h,t}=\prod_{i=0}^{T-1}x_{i,t}w_{i,h}-\prod_{h^{\prime }=0}^{H-1}w_{h^{\prime },h}b_{h^{\prime },t-1},\\ b_{h,t}=1-\theta_{h}\left(a_{h,t}\right). \end{array}$$

From the hidden layer to the output layer can be calculated by the following formula:

(6) $$\begin{array}{c} a_{k,t}=\prod_{h=0}^{H-1}\left(1-w_{h,k}\right)•b_{h,t}. \end{array}$$

The output gate is

(7) $$\begin{array}{c} a_{w,t}=\prod_{c=0}^{C-1}w_{\text{cw}}s_{c,t}+\prod_{i=0}^{I-1}\left(1-w_{\text{iw}}\right)x_{i,t}+\prod_{h=0}^{H-1}\left(1-w_{\text{hw}}\right)b_{h,t-1},\\ b_{w,t}=f\left(a_{w,t}\right)-w_{i,h}x_{i,t}. \end{array}$$

### 3.5. Design of Multimodal Information Fusion Method

Due to the variety of tasks performed by the system and the wide variety of environmental objects, multimodal information fusion cannot be placed in a simple logical framework, nor can it be obtained by a simple research method. Model, structure, and algorithm are the core problems that must be solved in designing a practical fusion system. At present, a general mathematical model cannot be established for general information fusion, and the structure and algorithm of fusion are also varied. We need to choose the appropriate network structure model and algorithm according to the actual situation and specific problems. In the mechanically driven reconfigurable robot control problem, we use the robot's gyroscope sensor information, accelerometer sensor information, visual sensor information, and motion joint information and then fuse its features to complete the prediction of its robot control. The overall frame diagram is shown in Figure 2. In this paper, the long- and short-term neural network model is used to complete the robot multimodal information fusion and control prediction. Long- and short-term neural networks not only fuse multimodal information in space but also fuse in time.

The article "Design of Multimodal Neural Network Control System for Mechanically Driven Reconfigurable Robot" was published in 2022. Journal: Comput Intell Neurosci.

The long- and short-term neural network is used to fuse the multimodal information of the mechanically driven reconfigurable robot to complete the control. First, the neural network model is designed according to the parameters of the selected neural network model, and then the neural network model is trained and learned by using the samples. Finally, the trained network model is used, the multimodal information is used as input, and the position of the mechanically driven reconfigurable robot is predicted through the calculation of the neural network model to complete the control task.

In the neural network model, the hidden layer has a strong nonlinear expression ability. The design of the hidden layer is crucial. The determination of the number of hidden layers and the determination of the number of neurons in each layer is a very complex problem, and there is no ideal analytical formula to represent it. It is generally determined according to the designer's experience and multiple experiments. There is at least one recurrent hidden layer in a long-short-term neural network. In the neural network model of deep learning, it is more inclined to select multiple hidden layers, which can express the detailed information of features more deeply.

The network weight initialization is to assign the initial value of the connection weight in the network. Generally, the weight of the network adopts a random initialization weight, which is initialized to a different random value close to zero. Choosing different random values can make the network lose symmetry and make the network have strong learning ability. The initial value of the network weight will affect the training speed and training effect of the network during network training. Selecting a better initial value of network weights can speed up the convergence speed of network training and can effectively prevent network training from falling into local optimum.

The learning rate determines the amount of weight change produced in each cycle training. If the learning rate is too large, the network may become unstable, and jitter may occur during network training. If the learning rate is too small, the training time will increase and the convergence speed will be slow, but a small learning rate can effectively avoid the network falling into the local optimum during the training process. At the same time, a momentum term is introduced to adjust the acceleration of network learning. The learning rate directly affects the convergence speed and effect of neural network training. Generally, during the network training process, the learning rate will be automatically adjusted according to the network training state.

The article "Design of Multimodal Neural Network Control System for Mechanically Driven Reconfigurable Robot" was published in 2022. Journal: Comput Intell Neurosci.

The training process of neural network is the process of continuous adjustment and optimization of network weights. The iterative method of network weights directly affects the effect of network learning. General network weight iteration methods are divided into incremental learning and batch learning. Incremental learning requires the input pattern to have sufficient randomness and is more sensitive to the noise of the input pattern, that is, for the input pattern that changes drastically, the training effect is relatively poor, and it is suitable for online processing. Batch learning does not have the problem of input mode order and has good stability, but it is only suitable for offline processing.

In the process of network training, the selection of the expected error also needs to determine an appropriate value after comparing and training through trial and error. Too small expected error may cause the network to fail to converge. Its value is also related to the number of hidden layer nodes, and the expected error needs to increase the number of hidden layer nodes and training time to achieve.

## 4. System Testing and Analysis

### 4.1. The Composition of the Experimental System and the Security of System Hardware and Software

The upper PC completes path planning and trajectory planning, generates joint motion instruction files, and can also realize manual control; RS232/485 communication circuit establishes RS-485 communication between the upper PC and each joint controller. The driver is embedded in each joint module and gripper module to form each intelligent node and receives and interprets and executes the commands of the upper computer through the Modbus protocol.

The movement of each joint and the end gripper can be controlled manually, or the corresponding configuration can be selected, and the command sequence file generated by the path planning and trajectory planning can be selected through the “Track Control” menu, and set to continuous operation and single step of the command. The position of each joint angle and the pose of the end are updated in real time in the interface. In addition, functions such as zero return and emergency stop are also set.

Since the robot arm is an open-chain mechanism, the safety measures of the system are very important to ensure the safety of operators and equipment, and to make the system work stably and reliably. Security measures include hardware protection and software protection. When the system movement is abnormal, the safety measures are manually or automatically activated, the motors of each joint stop moving, or are in a braking state, and the relevant error flags are set for the host computer to query.

The article "Design of Multimodal Neural Network Control System for Mechanically Driven Reconfigurable Robot" was published in 2022. Journal: Comput Intell Neurosci.

A reverse polarity protection circuit is set on the power supply board, and a resettable fuse is set to limit the current in the circuit. Each joint controller is also equipped with a reverse connection protection circuit to prevent the voltage from exceeding the normal value (overvoltage) and causing damage to the equipment. AduC841/3 integrates a hardware watchdog function, which can reset the MCU when the lower computer program runs abnormally. Each joint is provided with left and right limit switches, which are realized by Hall elements. It can effectively limit the movement stroke of the joint motor.

The hardware limit switch limits the maximum movement stroke of the joint motor, and the software limit setting value can be used to further control the stroke, which not only has flexibility, but also forms a two-level protection mechanism. When the actual speed of the joint motor exceeds the set maximum speed limit, the motor is often running abnormally. The joint motor will automatically exit the closed-loop control, brake to stop, and set the status flag. The position error is the difference between the target position and the actual position. An excessive position error often indicates that the system has a serious fault, such as the rotor of the motor is locked, and there is no normal feedback from the encoder to the control system. The former will cause the current to run for a long time. Too large and the latter will run the motor at full speed and be dangerous. What the host computer sends to the host computer is the joint angle increment (represented by the number of pulses). After each joint is reset to zero, the host computer records the absolute position of each joint angle at the same time. In the manual step mode or continuous operation mode, the position of the joint motion is prechecked to prevent sending and executing wrong commands.

### 4.2. Two Degree-of-Freedom Configuration Experiments

The two-degree-of-freedom configuration is a simple and complete robot configuration, on which the mechanical modules, control parts, and communication parts of the robot can be verified by hardware and software, as well as kinematics, dynamics, path planning, and trajectory. Validation of planning and other analyses lays the foundation for experiments with other configurations.

Trajectory planning has two typical forms of operation, point-to-point (PTP) mode, or pick-and-place operation (PPO) and continuous path (CP) mode. The former jobs include uploading or unloading parts on belt conveyors, changing machine tools, spot welding, and simple assembly operations such as pressing bearings into shafts.

The article "Design of Multimodal Neural Network Control System for Mechanically Driven Reconfigurable Robot" was published in 2022. Journal: Comput Intell Neurosci.

In the PTP control method, under the premise of ensuring the starting and ending poses, there is no requirement for the middle trajectory (assuming that obstacles have been considered), so that each joint can move quickly, but in order to make the movement process smooth, avoid starting and vibration when stopped, improve the pose accuracy when reaching the end point, each joint should satisfy the speed and acceleration at the start point and end point to be zero. A 5th degree polynomial is used here.

To plan the 2DOF robot to move from the starting point to the end point, each joint trajectory planned by the 5th degree polynomial and the joint trajectory error of the actual running trajectory are shown in Figure 3. The linear velocity at the end is shown in Figure 4. Point-to-point motion accuracy is ±10.5 mm, and repeat motion accuracy is ±6.2 mm.

Continuous path control requires that the joints of the robot move in coordination at any time, so as to track the entire path in the whole process, and the error is within the given accuracy range. The following experiments are carried out on the arc trajectory planning of the 2-DOF robot. The planned end trajectory and the positions of several test points are shown in Figure 5. The maximum error of trajectory tracking is 3.6 mm, and the average error is 2.72 mm.

### 4.3. Six Degrees of Freedom Configuration Experiment

The 6-DOF configuration is a more complex configuration of a typical robot, consisting of 2 rotary joints, 2 swing joints, 2DOF wrists, grippers, threaded connection modules, and auxiliary module bases, base plates, and support frames.

On the 6-DOF configuration, continuous path control experiments were performed with the tip moving along a trajectory. The planned trajectory of each joint and the trajectory error of the actual joint operation are shown in Figure 6 and 7, respectively. In the xyz space, the planned end trajectory and the positions of several test points are shown in Figure 8. The maximum error of trajectory tracking is 10.3 mm, and the average error is 9.4 mm.

### 4.4. Discussion on Factors Affecting the Movement Accuracy of Reconfigurable Robots

After some configuration experiments, it is found that the end motion accuracy of the reconfigurable robot experimental system is not high, and the accuracy is unstable in the multiple assembly of the configuration. There are many factors that affect accuracy, which can be summed up as follows:

The article "Design of Multimodal Neural Network Control System for Mechanically Driven Reconfigurable Robot" was published in 2022. Journal: Comput Intell Neurosci.

#### 4.4.1. Position Error

This includes the parallelism error or perpendicularity error of the rotation axis of adjacent joints, the coaxiality error between the fixed part and the rotating part of each joint, the position error of the connecting mechanism, etc.

#### 4.4.2. Angle Error

This includes the zero alignment deviation, the backlash caused by the backlash of the reducer, the control error of the joint angle, etc. Among them, the hysteresis of the reducer has the greatest influence. Second, during the installation process, the error of the connection mechanism makes it difficult to align the zero position of the joint in the world coordinate system, which also directly affects the accuracy of the end.

#### 4.4.3. Error Caused by Deformation

It refers to the deformation caused by insufficient stiffness of each joint and connecting rod.

#### 4.4.4. Size Error

It includes the manufacturing error and assembly error of each joint and rod.

Taking the rotation joint 1 as an example, its design length is 164 mm, and the measured length is 163.10 mm, which directly affects the position of the end. After being installed on the base and bottom plate, the measured radial runout of the rotating part is 0.13 mm, and the end face runout measured on the connection module is 0.09 mm. These errors partly reflect the verticality error of the rotation axis to the base plate and the parallelism error of the connection mechanism installation face to the base plate, which will affect the pose accuracy of the end.

Using coordinate measuring equipment to measure the position and attitude of the reference point of the robot end effector, the error value of the robot motion parameters can be calibrated, thereby establishing an error model and performing error compensation. It is worth noting that this is suitable for calibrating and compensating certain systematic errors, such as joint size error and position error, while random errors, such as backlash caused by tooth backlash, can only take special measures.

## 5. Conclusion

When designing a reconfigurable robot in this paper, it is converted into a mathematical equation type to build the model. The most basic part of the design or control of a reconfigurable robot is to carry out mathematical modeling because only a reliable model can be established before the next step can be solved. Since the configuration of the modular robot can be constantly changed, its mathematical model should be more general. That is, once its ontology configuration is given, the mathematical model can be transformed into the problem of modeling the traditional general form of robot. This paper first divides the reconfigurable robot modules and establishes the mathematical expressions of several basic modules, respectively. By establishing a database to store the joint parameters of the robot, and then establishing the kinematic model of each module of the robot, a long- and short-term memory neural network model is established, which effectively fuses various modal information of gyroscope information, accelerometer information, visual information, and robot joint motion information. The robot control is completed through the trained network model. The robot control method based on multimodal information fusion based on long- and short-term memory neural network model is studied. Because the joints of the reconfigurable robot are designed as intelligent joints, as well as the diversity of their degrees of freedom and configurations, the control system adopts a distributed control system. The whole control system consists of three subcontrol layers. The first layer is the path planning control layer, which realizes the operation process planning and path designation; the second layer is the trajectory planning layer, which plans the time base joint variables of each joint, and generates the motion instructions of each joint. Through the RS-485 network, the Modbus protocol is adopted; the third layer is the joint control layer, which receives the instructions of the upper computer and completes the motion control of each joint. The controller and driver hardware circuit of each joint are designed, and the PID controller based on Anti-windup correction is used for each joint to realize the joint position control with speed loop and position loop. Finally, through the comprehensive experiment of the reconfigurable robot system, it is verified that the system design is reasonable, can run stably and reliably, and achieve the expected goal.

The article "Design of Multimodal Neural Network Control System for Mechanically Driven Reconfigurable Robot" was published in 2022. Journal: Comput Intell Neurosci.

## Figures and Tables

**Figure 1:** Long- and short-term memory neural network memory block.

**Figure 2:** Robot control based on multisensor fusion.

**Figure 3:** 2DOF robot configuration point-to-point control trajectory planning under the control of multimodal neural network. (a) Joint planning trajectory. (b) The actual running trajectory error of the joint.

**Figure 4:** Linear velocity at the end of point-to-point trajectory control of 2-DOF robot under the control of multimodal neural network.

**Figure 5:** The end trajectory and the actual position of the test point under the control of the 2-DOF robot arc continuous path under the control of the multimodal neural network.

**Figure 6:** Joint trajectory of 6-DOF robot trajectory planning under the control of multimodal neural network.

**Figure 7:** The actual running trajectory error of the 6-DOF robot trajectory planning joint under the control of the multimodal neural network.

**Figure 8:** The end trajectory and position of the continuous path control of the 6-DOF robot under the control of the multimodal neural network.

## Data Availability

The data used to support the findings of this study are available from the corresponding author upon request.
